The article "Cognitive Therapy for Children with Intellectual Disabilities: A New Look at Social Adaptation Skills and Interpersonal Relationships" was published in 2023. Journal: Occup Ther Int.

# Cognitive Therapy for Children with Intellectual Disabilities: A New Look at Social Adaptation Skills and Interpersonal Relationships

**DOI:** 10.1155/2023/6466836

**Published:** 2023-04-03

**Authors:** Gulnaz Kulnazarova, Zhamiliya Namazbaeva, Laura Butabayeva, Lazzat Tulepova

**Affiliations:** Department of Special Education, Abai Kazakh National Pedagogical University, Almaty 050010, Kazakhstan

## Abstract

The purpose of the study is to consider the factors influencing the development of the culture of interpersonal relationships and the effectiveness of the influence of cognitive therapy on improving social adaptation skills. The method of cognitive therapy included several types of activities. The first type of activities included group sessions, during which the weaknesses of the interaction and their correction were identified. The second type was conducted in the format of teaching standard models of interaction between people. The third type of activity aimed to teach children to build a dialogue with each other and express their desires and emotions. Classes were held 3 times a week throughout the year. The study was attended by pupils of 5-7 grades of Zhanuya boarding school and special correctional boarding school No. 7 for children with intellectual disabilities. The results of a randomized study demonstrated an increase in the indicators of teamwork skills, self-control, emotional stability, and independent decision-making. The indicators of cheerfulness, openness, sociability, and logical thinking also improved. But the factor of antisocial behavior decreased. All of these indicators directly affect socialization. This strategy can be applied in practice in various specialized boarding schools and schools for children with intellectual disabilities.

## 1. Introduction

The study of the behavior of children with intellectual disabilities is a rather relevant topic today. A decrease in intellectual abilities can occur due to various diseases and factors. The basis of pathogenesis is central nervous system disorders [1]. These can be chromosomal pathologies such as Down, Patau, and Edward syndromes. Also, chromosomal abnormalities include Angelman syndrome and Prader-Willi syndrome. The features of chromosomal abnormalities include not only delayed intellectual development but also somatic abnormalities. These include sinistral immunity, visual problems, and abnormalities of the nervous system [2]. Abnormalities in mental development can also occur due to complications during pregnancy and childbirth, as well as due to external factors, for example, if the mother had TORCH infections during pregnancy or was exposed to high ionizing radiation doses. Quite often, birth trauma and fetal asphyxia can be the causes of developmental delay. A negative factor can be the mother's use of alcohol and drugs during pregnancy [3]. Also, a decrease in the level of intelligence is observed in the absence of proper education and training of children in their first years of life, this often happens in dysfunctional families [4]. These children often have communication problems with the people around them. First, due to a decrease in intelligence, children are not always able to formulate and express their thoughts clearly, which often leads to misunderstandings [5]. Secondly, emotional adaptation is impaired, which is characterized by the inability of children to adequately respond to various situations and can also be manifested through isolation and avoidance of social contacts [6]. Due to these factors, most children with intellectual disabilities have problems with socialization and self-realization in society. To help these children, programs are often used to develop their social and communication skills. They are usually implemented at specialized schools [7]. Due to the fact that the problem is global, there are quite a lot of options for such training. Various cognitive behavioral practices are very often used to teach interpersonal relationships [8]. For example, there are real-time play therapy techniques: each participant must build a dialogue and learn to solve various problems together with another person or a group of people under the supervision of a teacher or psychologist [9]. Cognitive therapy options using various mobile applications are also being considered. These can be simple games with cards that help children communicate with others and by choosing one or another card, to show their emotions and desires. This makes it easier to understand the needs of children [10]. There are applications that simulate certain situations, teach reactions, and, through repetition, reinforce the acquired skill. For example, there are mobile phone applications that match a word to an object or colour [11]. Currently, consideration is being given to introducing a virtual universe using computer technology. This makes it possible to expand the variability of tasks and enhance visual fixation during trainings [12]. Despite the positive dynamics and all possible options for the socialization of children with intellectual disabilities, it should be borne in mind that most studies have certain gaps. Many of them require additional research in various focus groups to obtain new results [13]. The problem of the culture of relationships among people with intellectual disabilities is quite relevant. Their inability to build social relationships reduces the quality of life and prevents them from becoming full-fledged members of society. Therefore, new training and psychological assistance programs are constantly being developed in the world. This not only provides an opportunity for socialization but also helps to change the attitude of society towards people with impaired intellectual functions. More research is required to understand the effectiveness of the impact of cognitive techniques on interpersonal culture. It is necessary to introduce similar experimental methods in schools and boarding schools for children with intellectual disabilities.

The article "Cognitive Therapy for Children with Intellectual Disabilities: A New Look at Social Adaptation Skills and Interpersonal Relationships" was published in 2023. Journal: Occup Ther Int.

## 2. Literature Review

Scientists from Sydney (Australia) conducted research on impaired social interaction skills among children with intellectual disabilities. They concluded that the main problem lies in the impairment of the neuropsychological profile as such children often have affective and comorbid disorders. This leads to impaired memory, learning, and expression of one's own thoughts and emotions. In most cases, attention deficit hyperactivity disorder occurs. Due to this, communication becomes difficult. It was also concluded that there are very few methods for helping such children and the best choice is cognitive behavioral therapy. However, the data on the effectiveness of the influence turned out to be rather controversial [14]. There was an experiment conducted in the UK to introduce cognitive programs to help people with congenital disabilities. The concept was to learn to distinguish between behaviors, thoughts, feelings, and emotions and to relate them to different situations. It was a randomized study involving people with mild to moderate mental retardation. These training sessions significantly improved understanding of one's own emotions, as well as the ability to respond correctly to various life situations [15]. Swedish researchers considered the impact of cognitive group training on the socialization of children with autism spectrum disorders. As part of the experiment, the effectiveness of this method has been confirmed [16]. Studies by South Korean researchers on the issue of socialization and improvement of communication skills among people with intellectual disabilities also confirmed their effectiveness. The methodology aimed to teach people the rules of communication, etiquette, and cultural characteristics of the region. An intragroup study demonstrated a fairly high efficiency [17]. In Victoria (Australia), researchers considered the effects of cognitive behavioral therapy on the social skills of children and adolescents. A randomized experiment, which confirmed the positive impact of behavioral interventions on children with socialization deficits, was carried out [18]. Scientists from Maribor (Slovenia) considered play intervention for children with developmental disabilities. All games were built on the development of cognitive skills, fine motor skills, social skills (adequate interpretation of emotions), and expansion of vocabulary. All games were played in a digital environment. The experiment studied children with autism and attention deficit disorder. However, the results were controversial. While the serious play method reduced anxiety and stress indicators and contributed to the recognition and management of emotions, clinical evidence of the benefits of this strategy was not revealed [19]. In Ireland, a strategy for the development of communication and language skills in children with Down syndrome was considered. The study said that the development of the social abilities in these children should start at a very early age. This is associated with the fact that contact and communication with people around them affects the level of communication skills of people with a similar disorder. Thus, it was concluded that social skills should be improved not only by the teacher but also by the parents or guardians. This requires that parents are taught to find contact with their children [20]. Indian researchers have studied the preoccupation with activities in children with intellectual disabilities. The experiment involved two focus groups, one of which consisted of absolutely healthy children, and the second one included children with various types of intellectual disabilities. The researchers let the children play in the classroom with ordinary toys (construction kits, figurines, cars, dolls) and watched the process. As a result, they noticed that the immersion and enthusiasm of children with mental disabilities in the game is much higher than that of healthy children. This should be taken into account as a psychological feature of children with intellectual disabilities in order to properly select a correction program [21]. Based on the data obtained, some conclusions can be drawn about teaching communication skills to people with intellectual disabilities. First, it should be borne in mind that the main socialization problems mainly occur due to the presence of comorbid and affective disorders. It should be taken into account that earlier development will determine the effectiveness of the selected strategy. Secondly, there is a need to choose the right approach for these children. One of the best options is cognitive therapy. There are a lot of cognitive therapy options: from individual sessions with a specialist to ready-made mobile applications and computer games. Thirdly, it is worth noting that most of the experiments are randomized studies. Therefore, precisely accurate results cannot be confirmed and such strategies require further research.

The article "Cognitive Therapy for Children with Intellectual Disabilities: A New Look at Social Adaptation Skills and Interpersonal Relationships" was published in 2023. Journal: Occup Ther Int.

### 2.1. Setting Objectives

The motivation is to conduct more studies on the impact of cognitive therapy on the culture of interpersonal relationships among children with intellectual disabilities to understand the degree of effectiveness. Cognitive therapy has not yet been completely studied, and more research is needed. In the course of the study, it is also worth finding out in which areas this technique can be applied and how appropriate it is. The main goal was to study the influence of cognitive behavioral therapy on the socialization of children with intellectual disabilities aged 11-13. A randomized study was conducted at specialized (correctional) boarding school No. 7 and Zhanuya boarding school. A total of 350 children took part in the study. The objectives included the introduction of cognitive therapy in the education of children with intellectual disabilities. Also, to clarify the degree of socialization problems and test the effectiveness, specialized testing was used to assess communicative competence. This test was implemented to evaluate the effectiveness of the integrated methodology. Further prospects of using the cognitive therapy strategy were also assessed. Specialized testing was used to analyze progress in the study. This was carried out and evaluated by a specialist in psychology.

## 3. Methods

### 3.1. Research Design and Sample

A randomized study was conducted to assess the impact of cognitive behavioral therapy on children with intellectual disabilities. This study looked at the uncontrolled before-after design. There was no control group in the study. The experiment involved students of specialized boarding school No. 7 and Zhanuya boarding school (Almaty). These were 5-7 grade students. The age of the respondents was 11-13 years old. The experimental group consisted of 350 participants. There were 180 boys and 170 girls among the respondents. The objectives of the experiment were to introduce cognitive therapy into the education of children with intellectual disabilities. A specialized test to assess communicative competence was also used to clarify the extent of socialization problems and to verify effectiveness. This questionnaire was administered to evaluate the effectiveness of the comprehensive methodology. Further perspectives of the cognitive therapy strategy were also evaluated. Specialized testing was used to analyze the progress of the study. It was conducted and evaluated by a specialist in psychology. Outside the study, the children attended school in accordance with their timetable. No additional psychological therapy was performed.

The article "Cognitive Therapy for Children with Intellectual Disabilities: A New Look at Social Adaptation Skills and Interpersonal Relationships" was published in 2023. Journal: Occup Ther Int.

### 3.2. Experiment

Prior to the experiment, all respondents were tested to evaluate their communicative and social competence. This is a multifactorial questionnaire that makes it possible to assess the position of the individual in society and make a probable forecast of their further social activity. It includes 100 questions and the assessment of such criteria as factor A (openness, sociability), factor D (assessment of cheerfulness), factor K (desire to work in a team), factor P (propensity for antisocial behavior), factor M (independence and independence of other people's opinions), factor N (self-control), and factor V (developed logical thinking). Each indicator is assessed on a 20-point scale except for factor P that is evaluated on a 40-point scale. Psychometric properties of this test include reliability (0.94-0.90), validity (0.85-0.8), and discriminability (0.33) [22]. The participants were tested at the beginning, in the middle, and at the end of the study. The experiment took place over four months. The therapy sessions were carried out 3 times a week. Each session lasted 3 hours. All training sessions were conducted under the guidance of a psychologist and a supervisor. Each of the three sessions that were carried out during the week had its own specifics. As part of the first type of training, collective therapy aimed at identifying the weaknesses of the interaction and their correction was carried out. This involved group sessions. Thus, a small group of children was selected to find a way out of a simulated situation through interaction with each other and teamwork. All respondents had to solve at least one case problem, after which they had to tell what emotions they experienced and analyze them [23]. The second type of activity was held in a training format. The children were shown standard models of interaction between people in various situations and had to repeat them to consolidate the material while acting out the scenario with each other [9]. The third type of session aimed to teach children to build a dialogue with each other by expressing their emotions and requests with the simulation of certain situations [24]. During these sessions, the respondents were divided into pairs. At the end of each month of the experiments, groups and pairs were disbanded and new ones were created to increase the level of adaptation of the respondents.

### 3.3. Statistical Processing and Data Analysis

The analysis was carried out using a questionnaire on communicative and social competence. It is a multifactor questionnaire which includes a measurement on eight criteria. The test itself consists of 100 questions. Seven of the criteria were assessed on a scale of 0 to 20 points, and only factor P (propensity for antisocial behavior) was assessed on a 40-point scale. Psychometric properties of this test include reliability (0.94-0.90), validity (0.85-0.8), and discriminability (0.33) The multifactor questionnaire is validated by Nikolai Petrovich Fetiskin (vice president of the International Academy of Psychological Sciences). This questionnaire was administered to all respondents three times: before the experiment, in the middle (interim testing), and at the end of the study.

The article "Cognitive Therapy for Children with Intellectual Disabilities: A New Look at Social Adaptation Skills and Interpersonal Relationships" was published in 2023. Journal: Occup Ther Int.

To process the data of this study, a specialized program for statistical analysis SPSS 26.0 was used. The results were interpreted and visualized with the help of the Microsoft Excel 2019 software package. Student's *t*-test was used to compare the effectiveness of the proposed teaching approach. To compare the mean result of the initial test with the results of the posttest to identify significant differences in the learning process. The level of significance was set at (*p* ≤ 0.05). 95% confidence intervals (CI) were calculated for median analysis.

### 3.4. Research Limitations

It should be noted that the degree of intellectual disability was not taken into account; all children were treated equally during the experiment. However, it should be taken into account that due to the varying degrees of intellectual disability, this therapy may not affect the participants in the same way. Also, the disease, which led to intellectual impairment, and its specificity were not taken into account. The experiment involved children with various pathologies. It should be noted that this is a completely randomized trial, the purpose of which is to determine the impact of cognitive behavioral therapy on the socialization of children with intellectual disabilities and teaching them communication skills. The results of the study will be considered in terms of the arithmetic mean of the sample. All these factors should be taken into account when considering the results of the experiment. It should also be noted that the study was not carried out after the experiment had ended. It is therefore not possible to say with certainty that the result remains at a static level.

### 3.5. Ethical Issues

Such experiments require the consent of the respondents. Due to the fact that the prospective participants have not yet reached the age of majority, the official decision can only be made by the persons responsible for them. Parents and guardians were informed verbally and in writing about the format of the experiment and all its details. After that, they gave their written consent for their children's participation in the study. The children gave their verbal consent to take part in the study after having been told about the essence of the experiment.

The article "Cognitive Therapy for Children with Intellectual Disabilities: A New Look at Social Adaptation Skills and Interpersonal Relationships" was published in 2023. Journal: Occup Ther Int.

## 4. Results

Before the experiment began, a communicative competence test was carried out. All the results of the respondents have an average value for the study group and are described as points and percentages. The preliminary result for factor A (openness and sociability) was 8 points (40%)—the lowest indicator of the average level of sociability. The result for factor D (cheerfulness) was 13 points (65%). The indicator of factor K (teamwork) turned out to be rather low -5 points (25%). Factor P (propensity for antisocial behavior) result was equal to 12 points out of 40 possible (30%). The score for factor M (independent decision-making) turned out to be rather low -6 points (30%). Factor N (self-control) also showed a low value of -5 points out of 20 possible (25%). Factor V (logical thinking) was equal to 4 points (20%). The result of factor C (emotional stability) is 6 points (30%), which is also a rather low indicator. The result is shown in Table 1.

Intermediate testing was carried out 2 months after the start of the experiment. The factor A results (openness and sociability) were 11 points (55%). This indicates an increase in sociability in the study group. In turn, factor D (cheerfulness) changed insignificantly; it increased by 1 point (70%). The factor K indicator (teamwork) increased by 3 points; thus, it was equal to 8 (40%). In two months, this indicator moved from the low level to the average level. Factor P (propensity for antisocial behavior) decreased to 10 points out of 40 possible (25%). The result of factor M (independent decision-making) increased to 9 points (45%). Factor N increased by two points and was equal to 7 points (35%). Logical thinking (factor V) also increased by 2 points and was equal to 6 points out of 20 possible (30%). Emotional stability (factor C) changed its value in a positive direction -8 points (40%). The result of intermediate testing is shown in Table 2.

At the end of the experiment, the final test was carried out. According to its results, factor A (openness and sociability) reached 13 points (65%). The factor D result (cheerfulness) was 15 points (75%)—the upper limit of the average level. Factor K (teamwork) amounted to 10 points (50%). The results of factor P (propensity to antisocial behavior) were equal to 8 points out of 40 (20%). The factor M indicator (independent decision-making) was 11 points (55%). The factor N indicator (self-control) was equal to 9 points out of 20 possible (45%). The result of factor V (logical thinking) was 8 points (40%). Factor C (emotional stability) reached 10 points (50%).

The article "Cognitive Therapy for Children with Intellectual Disabilities: A New Look at Social Adaptation Skills and Interpersonal Relationships" was published in 2023. Journal: Occup Ther Int.

The result of the final testing is shown in Table 3.

After the final test was calculated, it was compared with the preliminary results using Student's *t*-tests (Table 4). The significance level of A, K, and M is 0.008 (*p* ≤ 0.01). This result demonstrates the exclusion of the null hypothesis and acceptance of the alternative hypothesis. That is, it shows that there is a sufficient statistical difference between the “before” and “after” figures. The significance level of factor D is 0.005 (*p* ≤ 0.01). The significance level of factors P, V, and C is equated to 0.011 (*p* ≤ 0.05). And factor N has a significance level of 0.001 (*p* ≤ 0.001). It follows that all criteria underwent statistically significant changes in the course of the experiment.

Based on the data above, we can conclude that cognitive therapy sessions have a positive effect on the development of social skills in children with intellectual disabilities. This is evidenced by an increase in the indicators of teamwork, independent decision-making, self-control, logical thinking, and emotional stability. The criteria, such as “cheerfulness,” “openness,” and “sociability” also improved. It is worth noting that the factor of the propensity for antisocial behavior decreased due to the sessions of cognitive therapy. Also, changes in the behavior of the students who took part in the experiment began were noticed by their teachers. According to one of the supervisors, the children have really become more open in communication with each other and teachers, in particular. They are more actively involved in learning and open up to everything new with great interest. It is also worth noting that their academic performance has improved.

However, it should be considered that the study is completely randomized and was conducted in a large focus group. Also, the disease that provoked intellectual disability and its degree were not taken into account. Therefore, the absolute reliability of the results cannot be stated. In the future, additional research may be required.

## 5. Discussion

In 2019, a study on the thinking and behavior of children with intellectual disabilities was conducted in the Netherlands. The emphasis was placed on the assumption of the flexibility of behavior and personality factors. A randomized trial was conducted. The results showed that children with intellectual disabilities have more fixed thinking in terms of emotions and behavior. This suggests that teaching positive attitudes towards the development of the emotional sphere can be used to correct behavior and improve mental state [25]. It is impossible to fully compare this study with the present paper. This is due to the fact that the experiment, which was carried out in the Netherlands, does not involve cognitive therapy. However, the result obtained in the course of the Dutch research describes and confirms the positive dynamics that were obtained during the experiment described above in this study. In 2018, Canadian scientists conducted an experiment and studied the effect of cognitive behavioral therapy on the behavior of children with autism. The study was randomized. As a result, the scientists concluded that the indicators of emotional state and socialization skills improved in the focus group [26]. Comparing the results obtained by Canadian scientists with the results of this study, we can say that in both cases, there is a positive trend. The only difference is that in Canada, the focus group consisted exclusively of children with autism while this study looked at intellectual spectrum disorders more extensively. In 2018, there was an American study of the effect of cognitive therapy on children with self-regulation problems, namely, with social, executive dysfunction, and emotional spectrum disorders. The results proved the effectiveness of the impact of cognitive behavioral therapy on these areas of life [27]. This also confirms the feasibility of the application of this type of therapy to solve the problem of socialization in children with intellectual disabilities. Scientists from the UK have studied the effect of cognitive behavioral therapy on people with intellectual disabilities. They conducted a randomized trial. The results showed improved cognitive functions and improved quality of life [28]. The experiment by British researchers has confirmed the results of this study. Joint developments of scientists from China and the United States were based on studying the effectiveness of the use of cognitive therapy for resistance to various social situations in people with neurocognitive disorders. The results were ambiguous. Resistance to various social factors increased, but this did not affect neuropsychiatric behavioral symptoms [29]. However, the authors of this study argue that there could be various inaccuracies in the course of the experiment; therefore, absolute results cannot be claimed. Due to the fact that most studies in this area have positive dynamics, we can talk about confirmation of the effectiveness of this strategy, but it is also worth considering all the nuances associated with the design and conduct of these experiments. It is worth mentioning the fact that most studies are randomized; as a result of this, there may be certain gaps. It is impossible to identify the criteria for the effectiveness of the influence of cognitive therapy on people with certain disabilities as specific diseases and the degree of their development are not taken into account in most cases.

The article "Cognitive Therapy for Children with Intellectual Disabilities: A New Look at Social Adaptation Skills and Interpersonal Relationships" was published in 2023. Journal: Occup Ther Int.

The results obtained can be explained in terms of the fact that cognitive therapy is a learning factor. During the sessions, people work out new patterns of behavior reinforcing them by repetition. As people with various intellectual disabilities are able to learn the expression of various emotions and their manifestation in different situations, we can talk about an increase in acquired social skills.

The results described in this study are also randomized and cannot claim absolute accuracy; therefore, additional research is required in this area. During the comparison of this work with other articles, no fully similar methodology was found. It follows that this strategy may be a unique development.

The application of the knowledge gained gives us the understanding of the effectiveness of cognitive therapy in the development of a culture of interpersonal relationships in people with intellectual disabilities. This strategy can be used in the context of learning and developing social skills. This provides a prospect for new discoveries in the field of interpersonal relationships, as well as changing and improving the cognitive techniques aimed at people with a narrower specificity of intellectual disabilities.

However, it must be kept in mind that the degree of mental retardation was not taken into account; all children were treated equally in the experiment. Because of the varying degrees of mental retardation, the therapy may not affect the participants in the same way. The illness that led to mental retardation and its specifics were also not taken into account. Children with different pathologies participated in the experiment. This is a fully randomized study that aims to determine the effects of cognitive behavioral therapy on the socialization of children with intellectual disabilities and their learning of social skills. It should also be noted that the study was not carried out after the experiment had ended. It is therefore not possible to say with certainty that the result remains at a static level.

## 6. Conclusions

The results of this study showed that the use of cognitive therapy for the development of a culture of interpersonal relationships in children with intellectual disabilities has proven to be effective. This conclusion can be made based on the improvement of the indicators of self-control, teamwork, independent decision-making, logical thinking, and emotional stability. The indicators moved from the low level to the average one, which indicates an improvement in socialization skills. It is also worth noting a slight increase in the indicators of cheerfulness and sociability. The factor of antisocial behavior, in turn, decreased, which indicates a positive trend in the study. This leads to the conclusion that it is advisable to use cognitive therapy for the socialization of children with intellectual disabilities.

The article "Cognitive Therapy for Children with Intellectual Disabilities: A New Look at Social Adaptation Skills and Interpersonal Relationships" was published in 2023. Journal: Occup Ther Int.

The scientific value of this experiment lies in the applicability of the results for further research and the improvement of the methods of cognitive therapy in this area. It should be borne in mind that the study was based on a randomized sample method; therefore, this strategy requires additional experiments to obtain more accurate results. However, the method of cognitive therapy can be used to develop a culture of interpersonal relationships in people with intellectual disabilities. It should be used in schools and specialized institutions for children with intellectual disabilities. Also, the method of cognitive therapy can be used for preschool children with intellectual disabilities; however, it should be considered that this strategy may need to be adapted for this age group. Cognitive therapy can also help adults with intellectual disabilities socialize. Therefore, this strategy can be applied in private psychological practice.

When assessing the prospects for further research, it is worth pointing out the gaps in this research. The disadvantage is a rather large focus group of respondents, which does not give an absolute specificity of the results. It should be noted that due to the large number of participants, all results are considered in the mean value system. Also, intellectual disorders and the degree of their severity were not considered and were not taken into account. Standard cognitive therapy methods were chosen to promote socialization. Therefore, further research should examine the impact of such a strategy on a small group of respondents. Cognitive therapy to specific cases of intellectual disability, such as Down syndrome or autism, can also be applied. To obtain more accurate results, the sample should include respondents with the same severity of specific diseases. Other methods of cognitive therapy can also be applied. The results of such studies will make it possible to correct various cognitive methods in accordance with the degree and form of intellectual disabilities. This will contribute to the development of an individual approach and increased efficiency.

## Figures and Tables

**Table 1:** Preliminary results.

Name of factor	Points	Standard deviation	%
Factor A (openness, sociability)	8 points	1.3	40%
Factor D (cheerfulness)	13 points	1.6	65%
Factor K (teamwork)	5 points	1.2	25%
Factor P (propensity for antisocial behavior)	12 points	1.8	30%
Factor M (independent decision-making)	6 points	1.5	30%
Factor N (self-control)	5 points	1.1	25%
Factor V (logical thinking)	4 points	1.2	20%
Factor C (emotional stability)	6 points	1.4	30%

The article "Cognitive Therapy for Children with Intellectual Disabilities: A New Look at Social Adaptation Skills and Interpersonal Relationships" was published in 2023. Journal: Occup Ther Int.

**Table 2:** Intermediate results.

Name of factor	Points	Standard deviation	%
Factor A (openness, sociability)	11 points	1.1	55%
Factor D (cheerfulness)	14 points	1.4	70%
Factor K (teamwork)	8 points	1.2	40%
Factor P (propensity for antisocial behavior)	10 points	1.3	25%
Factor M (independent decision-making)	9 points	1.0	45%
Factor N (self-control)	7 points	0.8	35%
Factor V (logical thinking)	6 points	1.1	30%
Factor C (emotional stability)	8 points	1.0	40%

**Table 3:** Final results.

Name of factor	Points	Standard deviation	%
Factor A (openness, sociability)	13 points	0.7	65%
Factor D (cheerfulness)	15 points	0.6	75%
Factor K (teamwork)	10 points	1.1	50%
Factor P (propensity for antisocial behavior)	8 points	0.9	20%
Factor M (independent decision-making)	11 points	1.0	55%
Factor N (self-control)	9 points	0.7	45%
Factor V (logical thinking)	8 points	0.6	40%
Factor C (emotional stability)	10 points	0.9	50%

**Table 4:** Comparison of the results.

Scales	Preliminary results.	Final results	Empirical value	Significance level (*p* value)
Factor A	8 ± 0.141	13 ± 0.283	-22.361	0.008^∗∗^
Factor D	13 ± 0.141	15 ± 0.141	-14.142	0.005^∗∗^
Factor K	5 ± 0.283	10 ± 0.141	-22.361	0.008^∗∗^
Factor P	12 ± 0.141	8 ± 0.283	17.889	0.011^∗^
Factor M	6 ± 0.283	11 ± 0.141	-22.361	0.008^∗∗^
Factor N	5 ± 0.141	9 ± 0.141	-28.284	0.001^∗∗∗^
Factor V	4 ± 0.141	8 ± 0.283	-17.889	0.011^∗^
Factor C	6 ± 0.283	10 ± 0.141	-17.889	0.011^∗^

^∗^ *p* < 0.05; ^∗∗^*p* < 0.01; ^∗∗∗^*p* < 0.001.

## Data Availability

The data will be available on request.
